The article "Lessons from in vitro reconstitution analyses of plant microtubule-associated proteins" was published in 2014. Journal: Front Plant Sci.

# Lessons from *in vitro* reconstitution analyses of plant microtubule-associated proteins

**DOI:** 10.3389/fpls.2014.00409

**Published:** 2014-08-22

**Authors:** Takahiro Hamada

**Affiliations:** Department of Life Sciences, Graduate School of Arts and Sciences, The University of TokyoMeguro, Japan

**Keywords:** tubulin, microtubules, microtubule-associated proteins, MAPs, dynamic instability, plants, *in vitro* reconstitution analysis, Arabidopsis

## Abstract

Plant microtubules, composed of tubulin GTPase, are irreplaceable cellular components that regulate the directions of cell expansion and cell division, chromosome segregation and cell plate formation. To accomplish these functions, plant cells organize microtubule structures by regulating microtubule dynamics. Each microtubule localizes to the proper position with repeated growth and shortening. Although it is possible to reconstitute microtubule dynamics with pure tubulin solution *in vitro*, many microtubule-associated proteins (MAPs) govern microtubule dynamics in cells. In plants, major MAPs are identified as microtubule stabilizers (CLASP and MAP65 etc.), microtubule destabilizers (kinesin-13, katanin, MAP18 and MDP25), and microtubule dynamics promoters (EB1, MAP215, MOR1, MAP200, SPR2). Mutant analyses with forward and reverse genetics have shown the importance of microtubules and individual MAPs in plants. However, it is difficult to understand how each MAP regulates microtubule dynamics, such as growth and shortening, through mutant analyses. *In vitro* reconstitution analyses with individual purified MAPs and tubulin are powerful tools to reveal how each MAP regulates microtubule dynamics at the molecular level. In this review, I summarize the results of *in vitro* reconstitution analyses and introduce current models of how each MAP regulates microtubule dynamic instability.

## Introduction: microtubule structures and dynamics

Tubulin is a conserved GTPase in eukaryotes. Tubulin is classified into two major subfamilies, α- and β-tubulin, which form a rigid tubulin dimer. Tubulin dimers have two different states depending on whether β-tubulin is bound to GTP or GDP, similar to other GTPases. The GTP- and GDP-forms of the tubulin dimer are called GTP-tubulin and GDP-tubulin, respectively. GTP-tubulin, which is the active state, can polymerize into tubulin polymers that form a cylindrical filament up to 25 nm in diameter, the microtubule (Desai and Mitchison, 1997). Microtubules exhibit dynamic behavior, named “dynamic instability” *in vitro* (Mitchison and Kirschner, 1984; Horio and Hotani, 1986; Walker et al., 1988) and in cells (Cassimeris et al., 1988; Sammak and Borisy, 1988; Shelden and Wadsworth, 1993) with repeated growth and shortening at the tips (Figure 1). The dynamics of tubulin polymerization and depolymerization are explained by the GTP-cap model (Desai and Mitchison, 1997). Just after incorporation into the cylindrical microtubule, GTP bound by β-tubulin is hydrolyzed to GDP. Converted GDP-tubulin, which does not have polymerizing activity, starts to dissociate from the tip of microtubule. However, if another GTP-tubulin is attached to the tip, the dissociation of GDP-tubulin is repressed. In this model, the microtubule keeps growing as long as GTP-tubulin incorporation continues. When the incorporation of GTP tubulin stops, GDP-tubulins begin dissociating from the tip of the microtubule. The speed of shortening is about 100 times faster than the speed of growth. This transition is named “catastrophe.” Shortening microtubules occasionally start growing again. This transition is named “rescue” (Figure 1). Microtubule dynamics, including growth, shortening, catastrophe, and rescue, were also observed in plant cells (Shaw et al., 2003). Although plant cells have unique plant microtubule structures and organization processes (Hamada, 2014), microtubule dynamics are common in eukaryotes.

The article "Lessons from in vitro reconstitution analyses of plant microtubule-associated proteins" was published in 2014. Journal: Front Plant Sci.

**Figure 1:** **Illustration of microtubule dynamics**. A microtubule shows dynamic instability repeating growth and shortening. GTP-tubulin and GDP-tubulin were shown as colors of β-tubulin, yellow and green, respectively.

Microtubule dynamics based on tubulin polymerization and depolymerization can be accomplished by only the GTPase activity of tubulin. However, in cells, microtubules are surrounded by various proteins that regulate microtubule dynamics, functions, and structure formation. These proteins are named microtubule-associated proteins (MAPs). Therefore, the characterization of each MAP is important to understand microtubule dynamics in cells. Mutant analyses are powerful methods for clarifying how each MAP functions in plant cells. In plants, various mutants of MAPs have been obtained and their importance and essential roles have been described (Buschmann and Lloyd, 2008; Sedbrook and Kaloriti, 2008). On the other hand, mutant analyses give us limited information on how each MAP functions in microtubule dynamics at the molecular level. This limitation is mainly caused by the robustness of microtubule systems, which seem to be maintained by many species of functionally redundant MAPs. In fact, there are many reports that knockdown or loss of function mutants do not have a significant phenotype.

One method of analysis that complements the deficiencies of mutant analyses is “*in vitro* reconstitution analysis.” *In vitro* reconstitution analyses can examine precisely how each MAP changes microtubule dynamics under unique conditions in the presence of only that particular MAP and microtubules. Many reviews in the field of plant microtubules and MAPs have reported the results of mutant analyses and microtubule dynamics observations in cells; this review focuses on *in vitro* reconstitution analyses and introduces deduced plant MAP functions and mechanisms together with knowledge of yeast and animal MAPs.

The article "Lessons from in vitro reconstitution analyses of plant microtubule-associated proteins" was published in 2014. Journal: Front Plant Sci.

## *In vitro* reconstitution of tubulin dynamics

GTP-tubulin itself polymerizes into microtubules *in vitro* and in cells. In *in vitro* reconstitution experiments on tubulin dynamics, the amount of polymerized microtubules is generally analyzed rather than the tubulin GTPase activity, i.e., how much and how fast GTP is hydrolyzed to GDP. The amount of polymerized microtubules is dependent on the behavior of each microtubule (Desai and Mitchison, 1997). As described in the introduction, each microtubule independently exhibits dynamic instability, with repeated growth and shortening. Therefore, four parameters of microtubule dynamic instability (growth rate, shortening rate, catastrophe frequency, and rescue frequency) control the amount of polymerized microtubules.

Microtubules also show a pause state, which keeps the length of the microtubule constant, both *in vitro* and in cells. In most cases, the pause state is caused by balanced tubulin incorporation and dissociation at the microtubule tip, meaning that the pause state is a dynamic state rather than a static state. One exception is that some specific MAPs, such as the γ-tubulin complex at the minus end of the microtubule, inhibit tubulin incorporation and dissociation at the tip of the microtubule. During *in vitro* reconstitution experiments in the absence of capping MAPs, the pause state can be combined with the growth rate.

The idea of balanced tubulin incorporation and dissociation is also important for understanding the mechanism of microtubule dynamics and MAP functions. Microtubules are usually composed of 13 protofilaments and it seems that tubulin incorporation and dissociation occur at each protofilament independently. Following this idea, experiments using optical tweezers revealed that microtubules increase and decrease their own length at the nanometer scale during the growth and pause phases (Kerssemakers et al., 2006; Schek et al., 2007).

The dynamic instability of microtubules in *in vitro* reconstitution experiments is affected by the experimental conditions, such as tubulin concentration, GTP to GDP ratio and their concentrations, temperature, total ion concentration, and divalent cation species and their concentrations (Table 1). The amount of microtubules is increased when conditions are close to optimal, as all dynamic instability parameters tend to promote microtubule assembly. Conversely, the amount of microtubules is decreased when moving away from optimal conditions, as all dynamic instability parameters tend to promote microtubule disassembly. For example, an increase of tubulin concentration, which increases the amount of microtubules, leads to an increase of growth rate, a decrease of shortening rate, promotion of rescue frequency and suppression of catastrophe frequency. These observations fit well with the GTP cap model.

The article "Lessons from in vitro reconstitution analyses of plant microtubule-associated proteins" was published in 2014. Journal: Front Plant Sci.

**Table 1:** **Effects of experimental conditions on microtubule dynamics**.

**Conditions and agents**	**Amount of microtubules**	**Growth rate**	**Shortening rate**	**Catastrophe freq**.	**Rescue freq**.
Increase tubulin concentration (Walker et al., 1988)	Increase	Increase	Decrease	Decrease	Increase
Decrease tubulin concentration (Walker et al., 1988)	Decrease	Decrease	Increase	Increase	Decrease
GDP (Vandecandelaere et al., 1995)	Decrease	Decrease	Decrease	Increase	N. S.
Calcium ion (O'Brien et al., 1997)	Decrease	N. S.	Increase	Increase	Decrease
Nocodazole (Vasquez et al., 1997)	Decrease	Decrease	Decrease	Increase	N. S.

Amount of microtubules reflect the results of each parameter change of dynamic instability (Growth rate, Shorting rate, Catastrophe frequency, and Rescue frequency). The data of “Amount of microtubules” were determined by tubulin solution turbidly measurement of spectrophotometer or centrifugation sedimentation assay. Dynamic instabilities were measured from microscopy of each microtubule. N.S. means “Not Significant.”

Importantly, it is hard to compare different experimental data directly, especially from different laboratories and scientists, because a great number of factors affect microtubule dynamic instability, as described above. Strictly speaking, the qualities of tubulin and MAPs are sometimes different even if the same scientist prepares the proteins carefully. Therefore, in this review, I introduce general outlines of MAP characteristics in *in vitro* experiments without arguing the differences in detail.

## Microtubule stabilizers: Arabidopsis and tobacco MAP65 family and CLASP

Typical classical MAPs stabilize microtubules *in vitro*. These microtubule-stabilizing MAPs usually bind to the lateral side of microtubules and change the dynamic instability (Table 2). A change in only one parameter of dynamic instability is enough to increase the amount of microtubules.

**Table 2:** **Effects of microtubule stabilizers on microtubule dynamics**.

	**Amount of microtubules**	**Growth rate**	**Shortening rate**	**Catastrophe freq.**	**Rescue freq.**
Tau (Drechsel et al., 1992; Pryer et al., 1992; Trinczek et al., 1995)	Increase	Increase	Decrease	Decrease	Increase
MAP2 (Pryer et al., 1992; Kowalski and Williams, 1993; Itoh and Hotani, 1994)	Increase	Increase	Decrease	Decrease	Increase
cls1p, fission yeast (Al-Bassam et al., 2010)	Increase	Increase	Decrease	Decrease	Increase
MAP65-4, Arabidopsis (Fache et al., 2010)	–	N. S.	N. S.	Decrease	Increase
MAP65-2, Arabidopsis (Li et al., 2009)	–	–	–	Decrease against cold treatment	–
MAP65-1b, tobacco (Wicker-Planquart et al., 2004)	–	–	–	Decrease against cold treatment	–

*N.S. means “Not significant.” Minus signs represent “Not determined.” Measurement methods are described in Table 1 legend*.

The article "Lessons from in vitro reconstitution analyses of plant microtubule-associated proteins" was published in 2014. Journal: Front Plant Sci.

For example, animal neuronal MAPs, such as tau and MAP2, stabilize microtubules by lateral side binding (Drechsel et al., 1992; Pryer et al., 1992; Kowalski and Williams, 1993; Itoh and Hotani, 1994; Trinczek et al., 1995). Although there is some inconsistent data on how much each dynamic instability parameter contributes to microtubule stabilization, it is possible to summarize roughly that all dynamic instability parameters are turned in the direction of stabilizing microtubules. That is, these MAPs increase growth rate, decrease shortening rate, promote rescue frequency, and suppress catastrophe frequency.

In addition, it was recently reported that CLASP affects dynamic instability and stabilizes microtubules (Al-Bassam et al., 2010). CLASP accumulates at the microtubule tip through interaction between the CLASP CAP-Gly (cytoskeletal associated protein glycine-rich) domain and the plus tip accumulating protein, EB1. On the other hand, CLASP also has microtubule binding activity with a microtubule-binding domain, the TOG domain. Therefore, CLASP only binds to the lateral side of microtubules in the absence of EB1. *In vitro* reconstitution experiments using CLASP and purified tubulin have revealed that CLASP increases the amount of microtubule assembly by decreasing the shortening rate, promoting the rescue frequency, and suppressing the catastrophe frequency. The data clearly show that CLASP is a microtubule stabilizing MAP.

In plants, although homologs of tau and MAP2 have not been identified, many MAPs including CLASP bind to the lateral side of microtubules (Ambrose et al., 2007; Kirik et al., 2007; Hamada et al., 2013) and may stabilize microtubules to greater or lesser degrees. Some members of the MAP65 family, which have microtubule bundling ability with lateral side binding, have microtubule stabilizing activities. The clues of MAP65 microtubule-stabilizing activities were mentioned that microtubules bundled by tobacco MAP65-1b, Arabidopsis MAP65-1 and Arabidopsis MAP65-2 have resistance against cold-induced microtubule depolymerization, although these MAP65s do not promote microtubule assembly (Smertenko et al., 2004; Wicker-Planquart et al., 2004; Li et al., 2009). Fache and colleagues made great progress in analyzing the dynamic instability of each microtubule in microtubule bundles that were driven by Arabidopsis MAP65-4 (Fache et al., 2010). MAP65-4 stabilized the microtubules in the microtubule bundle by increasing the rescue frequency and reducing the catastrophe frequency. MAP65-4 did not affect either the growth rate or shortening rate.

The article "Lessons from in vitro reconstitution analyses of plant microtubule-associated proteins" was published in 2014. Journal: Front Plant Sci.

## Microtubule destabilizers: Arabidopsis kinesin-13, katanin, MAP18, MDP25

Some MAPs have the ability to destabilize microtubules and reduce the amount of microtubule assembly. To destabilize microtubules, MAPs need to change one or more parameters of dynamic instability in these directions: decreasing the growth rate, increasing the shortening rate, suppressing rescue frequency and promoting catastrophe frequency (Table 3).

**Table 3:** **Effects of microtubule destabilizers on microtubule dynamics**.

	**Amount of microtubules**	**Growth rate**	**Shortening rate**	**Catastrophe freq.**	**Rescue freq.**
XKCM1/kinesin-13, frog (Walczak et al., 1996)	Decrease	N. S.	N. S.	Increase	N. S.
Kinesin-13A, Arabidopsis (Oda and Fukuda, 2013)	Decrease	–	–	–	–
kip3/kinesin-8, Budding yeast (Varga et al., 2006)	Decrease	–	Increase	–	–
Kar3p/kinesin-14, Budding yeast (Endow et al., 1994)	Decrease				
Katanin, Sea urchin (McNally and Vale, 1993)	Decrease	–	–	–	–
katanin p60, Arabidopsis (Burk and Ye, 2002; Stoppin-Mellet et al., 2002)	Decrease	–	–	–	–
Stathmin, human (Curmi et al., 1997)	Decrease	Decrease	–	Increase	–
Stathmin, human (Howell et al., 1999)	Decrease	Decrease	Decrease	Increase	N. S.
Stathmin, human (Manna et al., 2006)	Decrease	Increase	N. S.	Increase	Inconsistent
MAP18, Arabidopsis (Wang et al., 2007)	Decrease	–	–	–	–
MDP25, Arabidopsis (Li et al., 2011)	Decrease	–	Increase	–	–

*N.S. means “Not significant.” Minus signs represent “Not determined.” Measurement methods are described in Table 1 legend*.

One of the microtubule destabilizing factors is the microtubule depolymerizing kinesin family (Moores and Milligan, 2006). Kinesin family members are motor proteins that move along microtubules by hydrolysis of ATP. Most kinesins function in organelle and protein transport along microtubules, but some have the unique ability to destabilize microtubules. The kinesin-13 family is the most famous microtubule-destabilizing kinesin group (Walczak et al., 1996; Desai et al., 1999). Kinesin-13 directly binds to the tips of microtubules and induces catastrophe (Desai et al., 1999; Helenius et al., 2006). Importantly, kinesin-13 can destabilize both taxol-stabilized and GMPCPP-stabilized microtubules. These taxol- and GMPCPP-stabilized microtubules do not show dynamic instability and also do not depolymerize in normal physiological conditions, indicating that kinesin-13 can remove GTP-tubulins from microtubule tips. The kinesin-13 family is also conserved in plants and it was proved that Arabidopsis kinesin-13A could ATP-dependently depolymerize microtubules (Oda and Fukuda, 2013).

The article "Lessons from in vitro reconstitution analyses of plant microtubule-associated proteins" was published in 2014. Journal: Front Plant Sci.

Besides kinesin-13, some proteins in the kinesin-8 and kinesin-14 families also have microtubule destabilizing activities *in vitro*. Kip3p, a member of the kinesin-8 family, accumulates at microtubule plus tips and destabilizes microtubules (Varga et al., 2006). Kip3p moves along microtubules to the plus end, which it specifically depolymerizes. Interestingly, the speed of kip3p-driven microtubule depolymerization is increased dependent on microtubule length, meaning that Kip3p translocation toward the plus end is important for microtubule depolymerization. The targeting mechanism in kip3p/kinesin-8 is unique because kinesin-13 is targeted to both the plus and minus ends of microtubules directly (Helenius et al., 2006). Kar3p, a member of the kinesin-14 family, was identified as a minus end-directed kinesin and specifically depolymerizes the minus ends of microtubules (Endow et al., 1994). However, Kar3p forms a heterodimer with the interacting protein Cik1p in cells. *In vitro* reconstitution analyses with Kar3p and Cik1p revealed that Kar3/Cik1 complexes move toward the plus ends of microtubules and destabilize them from the plus end (Sproul et al., 2005). Although obvious homologs of Kip3 and Cik1p have not been identified in plants, similar kinesins might exist because kinesins are very diverse in plants (Richardson et al., 2006).

Katanin is a microtubule-severing factor. Katanin p60/p80 heterodimer complexes accumulate around the microtubule and sever it at the surrounded region through ATP hydrolysis. Although it seems that katanin does not regulate microtubule dynamics directly, the exposed face of the microtubule after cutting by katanin often experiences catastrophe because the inside of microtubules is composed of GDP-tubulin. Thus, an increase of katanin proteins in *in vitro* reconstitution experiments led to a decreased amount of microtubule assembly (McNally and Vale, 1993). Katanin is conserved in plants and its microtubule-severing abilities were confirmed in *in vitro* reconstitution experiments (Burk and Ye, 2002; Stoppin-Mellet et al., 2002). The knowledge of katanin molecular mechanism in animal would be available in plants because there is no particular difference between them. Interestingly, the importance of katanin in plants is well characterized in mutants that have prominent phenotypes (Bichet et al., 2001; Burk et al., 2001; Webb et al., 2002; Bouquin et al., 2003). Loss of katanin activity causes excess stabilization of microtubules and inhibits the rearrangement of microtubules in plant cells.

The article "Lessons from in vitro reconstitution analyses of plant microtubule-associated proteins" was published in 2014. Journal: Front Plant Sci.

Chemical inhibitors of tubulin polymerization, such as colchicine, vinblastine, oryzalin and propyzamide, bind to tubulin dimers and inactivate tubulin even in the presence of GTP. Like these inhibitors, some proteins bind to tubulin dimers and inhibit tubulin polymerization. Animal stathmin/Op18, which binds to tubulin dimers, decreases the growth rate and promotes the catastrophe frequency in *in vitro* reconstitution experiments (Curmi et al., 1997; Howell et al., 1999). The effects of stathmin/Op18 on dynamic instability are similar when the tubulin concentration is decreased. However, in addition to tubulin inactivation, stathmin/Op18 also increases catastrophe by a different mechanism that directly affects microtubule ends (Howell et al., 1999; Manna et al., 2006; Gupta et al., 2013). These findings indicate that stathmin/Op18 favors protofilament structures and peels off tubulin dimers at the microtubule ends. In plants, MAP18 and MDP25 have been identified as microtubule destabilizers. These proteins have a typical microtubule binding domain with a cluster of hydrophobic residues (Wang et al., 2007; Li et al., 2011). In *in vitro* reconstitution experiments, MDP25 increased the shortening rate from 0.26 to 1.16 μm/min (Li et al., 2011). Interestingly, MDP25 destabilized taxol-stabilized microtubules, especially in the presence of calcium ions (Qin et al., 2012). It was reported that tubulin dimers often form protofilament-like structures in the presence of taxol and calcium ions (Elie-Caille et al., 2007). MDP25/MAP18 might prefer protofilament structures and peel off tubulin dimers from microtubule ends like stathmin/Op18.

## EB1 family: Arabidopsis EB1

The plus end is the most dynamic region of the microtubule and accumulates a great number of MAPs, called +TIPs. EB1 seems to be the most important +TIP because most +TIPs require EB1 binding to localize to the microtubule plus end (Kumar and Wittmann, 2012). EB1 labels only growing microtubules because it specifically recognizes tubulin protofilament sheets with tubulin dimers in the intermediate GTP hydrolysis state (Maurer et al., 2012). Although the accumulation of individual +TIPs depends on EB1 to influence microtubule plus end dynamics, EB1 itself can also change the dynamic instability of microtubules at the plus end.

The article "Lessons from in vitro reconstitution analyses of plant microtubule-associated proteins" was published in 2014. Journal: Front Plant Sci.

In *in vitro* reconstitution experiments, animal EB1 increased the amount of microtubules by increasing growth rate and rescue frequency (Table 4). In addition, unexpectedly, EB1 promoted the catastrophe frequency (Vitre et al., 2008; Komarova et al., 2009; Table 4). The paradoxical promotion of both growth rate and catastrophe frequency was explained by the sheet closure model (Vitre et al., 2008). In this model, accumulated EB1 at the tubulin sheet stimulates sheet closure and subsequent β-tubulin GTP hydrolysis, meaning that the short GTP cap often induces catastrophe. Increase of catastrophe frequency was also observed in the fission yeast EB1 homolog, Mal3 (Bieling et al., 2007) and resent works (Li et al., 2012; Zanic et al., 2013; Maurer et al., 2014). On the other hand, results of increase of catastrophe frequency by EB1 are still controversial because human EB1 decreased or did not affect catastrophe frequency (Manna et al., 2008; Dixit et al., 2009). It is still unclear whether this discrepancy was caused by differences in the nature of the proteins or experimental conditions. Further analyses are required to reach a conclusion.

**Table 4:** **Effects of microtubule dynamics promoters on microtubule dynamics**.

	**Amount of microtubules**	**Growth rate**	**Shortening rate**	**Catastrophe freq.**	**Rescue freq.**
EB1, mouse (Vitre et al., 2008)	Increase	Increase	Decrease	Increase	Increase
EB1, human (Manna et al., 2008)	Increase	Increase	Decrease	Decrease	Increase
EB3, human (Komarova et al., 2009)	Increase	Increase	Decrease	Increase	Increase
Mal3, fission yeast (Bieling et al., 2007)	Increase	Increase	Decrease	Increase	Increase
EB1a, Arabidopsis (Komaki et al., 2010)	Increase	–	–	–	–
XMAP215, frog (Gard and Kirschner, 1987; Vasquez et al., 1994)	Increase	Increase	Increase	N. S.	Decrease
XMAP215, frog (Shirasu-Hiza et al., 2003)	–	–	–	Increase	–
XMAP215, frog (Zanic et al., 2013)	–	Increase	Increase	Increase	–
TOGp, human (Charrasse et al., 1998)	Increase	Increase	–	–	–
MAP200, tobacco (Hamada et al., 2004, 2009)	Increase	Increase	N. S.	Increase	Increase
stu2p, budding yeast (Van Breugel et al., 2003)	Decrease	Decrease	N. S.	Increase	–
SPR2, Arabidopsis (Yao et al., 2008)	Increase	Increase	Inconsistent	Increase	Increase

*N.S. means “Not significant.” Minus signs represent “Not determined.” Measurement methods are described in Table 1 legend*.

Plants have obvious EB1 homologs. Arabidopsis EB1 increased the amount of microtubules *in vitro* (Komaki et al., 2010), indicating that it increases growth rate or rescue frequency or both. Measurements of dynamic instability with plant EB1s will contribute to our understanding of the general microtubule regulation mechanism of EB1.

The article "Lessons from in vitro reconstitution analyses of plant microtubule-associated proteins" was published in 2014. Journal: Front Plant Sci.

## MAP215 family: Arabidopsis MOR1, tobacco MAP200

The Xenopus homolog of the MAP215 family, XMAP215 was identified from Xenopus egg extracts as a factor that dramatically increases the amount of microtubules *in vitro* (Gard and Kirschner, 1987; Table 4). The unique feature of the MAP215 family is that it not only promotes microtubule assembly but also promotes microtubule disassembly. In *in vitro* reconstitution experiments, XMAP215 promotes both the growth rate and shortening rate dramatically (Vasquez et al., 1994). XMAP215 was also identified as a catastrophe-inducing factor that destabilizes GMPCPP-stabilized microtubules *in vitro* (Shirasu-Hiza et al., 2003), suggesting that the enhancement of microtubule disassembly is its true function, but not by exhausting available GTP-tubulin through significant promotion of growth rate. The *in vitro* activity of stu2p, a budding yeast MAP215 homolog, supports this suggestion (Van Breugel et al., 2003). Stu2p is a unique homolog that has half the protein length of animal and plant MAP215 family members. In *in vitro* reconstitution experiments, stu2p promotes the disassembly of microtubules by increasing the catastrophe frequency and reducing the growth rate. In recent *in vitro* experiments with recombinant protein, XMAP215 clearly increased both the shortening rate and catastrophe frequency, as well as increasing the growth rate (Zanic et al., 2013).

The MAP215 family is also conserved in plants. The plant homolog in Arabidopsis was first identified as a mor1-1 mutant, which have abnormal microtubule structures (Whittington et al., 2001). Like the animal MAP215 family, *in vitro* reconstitution experiments showed that the tobacco homolog, MAP200, increases the amount of microtubules (Hamada et al., 2004). In addition, MAP200 increases the growth rate, rescue frequency and catastrophe frequency (Hamada et al., 2009), indicating that plant homologs of the MAP215 family also have unique futures to promote both microtubule assembly and disassembly.

How does the MAP215 family promote both microtubule assembly and disassembly? Several models were proposed to explain this unique function. The major discrepancy between models is caused by differences in the roles of five TOG domains. The TOG domain is a tubulin-binding domain and one TOG domain can bind to one tubulin dimer *in vitro* (Slep and Vale, 2007). The length of each TOG domain and MAP215 protein is approximately 6 nm and 60 nm, respectively (Cassimeris et al., 2001; Al-Bassam et al., 2007; Slep and Vale, 2007), meaning that one animal or plant MAP215 family protein could bind to five or more tubulin dimers theoretically. Fitting with this prediction, XMAP215 and MAP200 form complexes with multiple tubulin dimers (Cassimeris et al., 2001; Hamada et al., 2004, 2009). On the other hand, the budding yeast homolog stu2p has four TOG domains with self-dimerization. Interestingly, stu2p holds one tubulin dimer surrounded by four TOG domains (Al-Bassam et al., 2006). Like stu2p, it was confirmed that one XMAP215 also binds to one tubulin dimer in some conditions (Brouhard et al., 2008).

The article "Lessons from in vitro reconstitution analyses of plant microtubule-associated proteins" was published in 2014. Journal: Front Plant Sci.

Recently, the importance of the 1st and 2nd N-terminal TOG domains has been the subject of focus. Inactivation of the 3rd and 4th TOG domains of full-length XMAP215 increased the growth rate similar to normal XMAP215 in *in vitro* reconstitution experiments (Widlund et al., 2011). Interestingly, truncated proteins with the 1st and 2nd N-terminal TOG domains (TOG12) of XMAP215 or MOR1 also increased the growth rate or amount of microtubules *in vitro*, respectively (Widlund et al., 2011; Lechner et al., 2012), suggesting that TOG12 acts as a microtubule polymerase at least. Furthermore, the mutations of three MOR1 mutant lines in Arabidopsis were in the N-terminal TOG domain (Whittington et al., 2001; Konishi and Sugiyama, 2003), indicating the importance of this domain. One of the MOR1 mutants, *mor1-1*, which was caused by the amino acid substitution mutation L174F, showed a slow growth rate and shortening rate (Kawamura and Wasteneys, 2008). An *in vitro* microtubule co-sedimentation assay with mutated MOR1 TOG12 truncated protein revealed that L174F resulted in high affinity for microtubules (Lechner et al., 2012), indicating that the proper affinity of the TOG domain is important for MAP215 family functions.

The MAP215 family also has unique features. Cryo-electron microscopy revealed that XMAP215 forms a very long tubulin filament at the tip of the microtubule (Kinoshita et al., 2001). MAP200 also forms very long doublet tubulin filaments especially in the presence of taxol (Hamada et al., 2009). In addition, XMAP215 radically increased the growth rate in the presence of taxol (Zanic et al., 2013). These data suggest that MAP215 family members promote tubulin protofilament extension. Another important feature is that one XMAP215 showed processive movements at both growing and shortening microtubule ends (Brouhard et al., 2008). These processive movements might be related to specific protofilament extension and shrinkage at the microtubule tip.

Based on the results described above, we can imagine a number of mechanistic models for how the MAP215 family promotes growth rate. For example, the MAP215 family might accelerate tubulin incorporation like an enzyme or a mold, or change the stability of extended protofilaments, or suppress nano-scale tubulin dissociation during the growth phase. Although the details of the mechanism are unknown, processive movements and protofilament extension seem to be the keys for growth rate promotion.

The article "Lessons from in vitro reconstitution analyses of plant microtubule-associated proteins" was published in 2014. Journal: Front Plant Sci.

In contrast, it is hard to develop a mechanistic model for how the MAP215 family promotes disassembly (catastrophe or shortening) because the models of catastrophe mechanisms in pure tubulin solution remain inconsistent (Bowne-Anderson et al., 2013). Brouhard et al. (2008) proposed a model in which XMAP215 holds tubulin dimers in the intermediate state between tubulin incorporation and dissociation. This model can explain XMAP215-enhanced microtubule assembly and disassembly. However, there are some observations that the model cannot explain. MAP200 repressed the catastrophe frequency when a small amount of GDP was added to the *in vitro* assay despite it basically increasing the catastrophe frequency in normal conditions (Hamada et al., 2009). In the presence of a small amount of GDP, the growth rate is suppressed even in the presence of MAP200, indicating that the higher growth rate and increase of catastrophe might be correlated.

Protofilament-like structures at the microtubule ends were observed when XMAP215 depolymerized GMPCPP-stabilized microtubules (Shirasu-Hiza et al., 2003). Similarly to the promotion of growth rate, protofilament extension might be important for catastrophe initiation. Irregular microtubule lattice arrangements might induce catastrophe without the loss of the GTP cap (Chrétien and Fuller, 2000; Hunyadi et al., 2005). Alternately, protofilament extension by MAP215 family members might change their curved structures to straight like microtubules and induce catastrophe as well as the loss of lateral protofilament binding (VanBuren et al., 2002, 2005; Margolin et al., 2011, 2012).

XMAP215 and MAP200 have slight differences in their effects on the shortening rate and rescue frequency (Table 4). XMAP215 dramatically promotes the shortening ratem but does not influence rescue frequency. In contrast, MAP200 increases the rescue frequency but does not affect shortening rate. This difference might be explained as follows. Although microtubules are composed of GDP-tubulin, it was reported that some GTP-tubulin remained in the microtubule lattice without hydrolysis (Dimitrov et al., 2008). Rescue events often occurred at the position of the remaining GTP-tubulin cluster. I expect the remaining GTP-tubulin in the microtubule lattice might decrease the shortening rate of microtubules. XMAP215 might incorporate tubulin dimers with precisely executed GTP hydrolysis, resulting in shortening rate promotion but no effect on rescue frequency. In contrast, MAP200 might incorporate some GTP-tubulins without GTP hydrolysis, and subsequently induce an increase of rescue frequency without changing the shortening rate. Although the difference between the two homologs seems to be explained here, it is still unclear whether the difference is caused by the nature of each homolog or the conditions of the *in vitro* reconstitution experiments described above.

The article "Lessons from in vitro reconstitution analyses of plant microtubule-associated proteins" was published in 2014. Journal: Front Plant Sci.

## SPR2 family: Arabidopsis SPR2, SP2L

Plants have another TOG domain-containing MAP family, the SPIRAL2 (SPR2) family, in addition to CLASP and the MAP215 family. SPR2 has one TOG domain at the N-terminus and increases the amount of microtubules *in vitro*. Interestingly, SPR2 and its homolog SP2L increase the growth rate, catastrophe frequency and rescue frequency *in vitro* (Yao et al., 2008; Table 4). Further *in vitro* analyses are required to reveal the molecular mechanism of how the SPR2 family changes dynamic instability, and the difference between MAP215 and SPR2.

## Future perspectives

In this review, I summarized the results of *in vitro* reconstitution experiments with purified proteins. These results clearly reveal each MAP character. However, some MAPs do not play the expected roles in cells because many numbers and various types of MAPs regulate microtubule dynamics cooperatively or competitively in cells. Reconstitution of intracellular microtubule dynamics *in vitro* is one of challenges of *in vitro* reconstitution experiments after characterizing individual MAPs properties.

The pioneer study is the combination of XMAP215 and kinesin-13, which mainly promote microtubule growth rate and catastrophe frequency, respectively (Kinoshita et al., 2001). In this assay, the combination of XMAP215 and kinesin-13 changed *in vitro* dynamic instability parameters close to physiological parameters in cells comparing with the presences of each MAP. Recently, synergistic effects of EB1 and MAP215 family on microtubule dynamics were well characterized (Li et al., 2012; Zanic et al., 2013; Maurer et al., 2014). EB1 and XMAP215 family promote microtubule growth rate with different mechanisms. Growth rates were dramatically increased in the presence of both proteins. In addition, advanced study tried to reconstitute intracellular microtubule dynamics with adding EB1 binding proteins, sentin, to EB1 and XMAP215 family (Li et al., 2012).

*In vitro* reconstitution experiments with several purified MAPs will provide results like no others and help our understanding of MAPs functions along with other experiments such as mutant analyses.

The article "Lessons from in vitro reconstitution analyses of plant microtubule-associated proteins" was published in 2014. Journal: Front Plant Sci.

### Conflict of interest statement

The author declares that the research was conducted in the absence of any commercial or financial relationships that could be construed as a potential conflict of interest.
